# Cardiovascular Disease Risk Factors, Musculoskeletal Health, Physical Fitness, and Occupational Performance in Firefighters: A Narrative Review

**DOI:** 10.1155/2022/7346408

**Published:** 2022-09-19

**Authors:** Jaron Ras, Denise L. Smith, Andre P. Kengne, Elpidoforos E. Soteriades, Lloyd Leach

**Affiliations:** ^1^Department of Sport, Recreation and Exercise Science, Faculty of Community and Health Sciences, University of the Western Cape, Cape Town, South Africa; ^2^Health and Human Physiological Sciences, Skidmore College, Saratoga Springs, NY, USA; ^3^Non-Communicable Diseases Research Unit, South African Medical Research Council, Cape Town, South Africa; ^4^Department of Medicine, Faculty of Health Sciences, University of Cape Town, Cape Town 7700, South Africa; ^5^Harvard T. H. Chan School of Public Health, Department of Environmental Health, Environmental and Occupational Medicine and Epidemiology (EOME), Boston, USA; ^6^Open University of Cyprus, School of Economics and Management, Healthcare Management Program, Nicosia, Cyprus

## Abstract

**Introduction:**

Firefighting is a strenuous occupation that requires firefighters to be in peak physical condition. However, many firefighters have risk factors for cardiovascular disease, impaired musculoskeletal health, and are not physically fit for duty, which all negatively impact their occupational performance. Therefore, the aim of this review is to determine the relationship between cardiovascular disease risk factors, musculoskeletal health, physical fitness, and occupational performance in firefighters.

**Methods:**

The electronic databases PubMed, SCOPUS, and Web of Science were searched online via the library portal of the University of the Western Cape. Publications and grey literature between the years 2000 to present were used. In total, 2607 articles were identified; after the removal of duplicates 1188 articles were then screened, and were excluded for not meeting initial screening criteria. The remaining 209 full-text articles were screened based on the inclusion and exclusion criteria, where 163 articles were excluded. Only studies that were quantitative were included. This left 46 articles that were then finally included in the current narrative review.

**Results:**

The current literature indicated that significant relationships existed between cardiovascular risk factors, musculoskeletal health, physical fitness, and occupational performance. The results indicated firefighters who were aged, obese, physically inactive, cigarette smokers, and unfit were at the highest risk for cardiovascular and musculoskeletal health complications, and unsatisfactory occupational performance. Musculoskeletal health complications significantly affected occupational performance and work ability and were related to physical fitness of firefighters. Most cardiovascular risk factors were related to physical fitness, and all physical fitness parameters were related to occupational performance in firefighters.

**Conclusion:**

The overwhelming evidence in the current review established that physical fitness is related to occupational performance. However, the relationship between cardiovascular risk factors and musculoskeletal health in relation to occupational performance is less clear and still understudied. Significant gaps remain in the literature.

## 1. Introduction

Firefighting is a strenuous occupation that places tremendous strain on the body, where firefighters are routinely exposed to life-threatening situations, severe temperatures, hazardous chemicals, and fumes [1, 2]. These severe conditions necessitate that firefighters wear personal protective equipment that is heavy and insulated, augmenting the physiological load already placed on the cardiovascular and musculoskeletal systems [3]. These types of strenuous working conditions cause high levels of chronic cardiovascular and physical strain, predisposing firefighters to cardiovascular disease, musculoskeletal injury, morbidity and in extreme cases, mortality [1, 4, 5]. Firefighters are, therefore, required to be in optimal physical conditioning to overcome many of these work-related challenges to their health [6–8].

Previous research indicates that amongst the emergency services, firefighters have the highest percentage of mortality (45%) due to sudden cardiac death (SCD), which is related to the presence of multiple cardiovascular disease (CVD) risk factors and low levels of physical fitness [1, 4, 5]. Current literature indicates that the majority of firefighters are either obese (63%) or physically inactive (49%) and unfit (27.1%), and engaged in poor dietary practices [9–14]. In addition, many of them were hypertensive (42%), smokers (21%), diabetic (15%), or had a muscular disorder (25%) [9–14]. The presence of multiple CVD risk factors substantially increased the cardiovascular strain, and negatively affected their cardiovascular fitness and occupational performance [3, 15, 16]. Musculoskeletal injuries amongst firefighters occurred most commonly in the fire station, and were due to trips, slips, or falls. Either while performing physical activities in the fire station or when responding to emergency situations, and occurred more frequently in aged, obese, and inactive firefighters [17, 18]. The lower limbs, back, and shoulders were the most common anatomical sites of injury and musculoskeletal disorders [17–21]. These injuries and disorders frequently caused chronic pain and inflammation, and decreased the work-ability of firefighters, and negatively affected their musculoskeletal health and occupational performance [17, 21, 22]. Cardiovascular disease and musculoskeletal health are significantly related to and affect the occupational performance of firefighters [9, 23–27]. Maintenance of physical fitness is an essential preventative tool not only in maintaining cardiovascular and musculoskeletal health but also in maintaining satisfactory occupational performance in firefighters [6, 28, 29].

There have been very few studies investigating the relationship between CVD risk factors, musculoskeletal health, physical fitness, and occupational performance in firefighters. Therefore, this narrative review will investigate the relationships between these variables in firefighters, and how these may affect the overall health, wellness, and performance of firefighters. The objectives are to examine the relationship between each of these key outcome variables independently, and to highlight gaps in the literature for future research. The authors hypothesise that there will be significant relationships between CVD risk factors, musculoskeletal health, physical fitness, and occupational performance in firefighters.

### 1.1. Understanding the Key Concepts in the Review

In the present review, CVD risk factors encompass all the metrics related to increased cardiovascular risk status or decreased cardiovascular health. These parameters include aging, obesity, hypertension, diabetes, dyslipidaemia (hypercholesteremia), cigarette smoking, physical inactivity, a poor diet, and heart rate variability (HRV) [30, 31]. Heart rate variability is the variation in the time interval between consecutive heartbeats in milliseconds [1, 32].

Musculoskeletal health encompasses all factors related to the reduced integrity of the musculoskeletal system, and includes acute and/or chronic injuries, musculoskeletal disorders, discomfort, and pain [33–35].

Physical fitness includes all the components of health-related physical fitness that refers to the ability to perform muscular work satisfactorily and includes cardiorespiratory fitness, body composition, muscular strength, muscular endurance, and flexibility [36]. All components of health-related physical fitness are linked to occupational performance in firefighters.

Occupational performance refers to the ability to perform one's job adequately, to the standards that are required in the specific occupation, which, in this case, refers to firefighting [37]. For firefighters, occupational performance includes the ability to perform core duties, such as hose drag, victim drag, equipment carry, door breaches, and ceiling breaches.

## 2. Methods

### 2.1. Literature Search Strategy

The following electronic databases were searched: PubMed, SCOPUS, and Web of Science. Grey literature included the Networked Digital Library of Theses and Dissertations. Only publications between the years 2001 to December 2021 were used. Keywords and medical subject heading (MeSH) terms were used in various arrangements according to the specific database searched. An example of a search string used for a database search can be seen in Table 1:

### 2.2. Graphical Bibliography of Literature Search

Figure 1 explains the search results from PubMed, SCOPUS, and Web of Science as a diagram. The search results were saved and exported to Zotero™, where references were checked for duplicates. Thereafter, the citations were exported to VOSviewer™ where the bibliographic analysis was conducted. The diagram explains the central themes of the study, which were identified during the literature search procedure. The diagram indicates the commonly used terms, keywords, themes, and subthemes in the various articles from the electronic databases and their association with each other. The diagram was normalized using LinLog/modularity. The size of the node and line width between nodes indicates the commonality and popularity of the search terms, keywords, and co-occurrences. The co-occurrence and network strength of the keywords are represented by the size of the node and the degree of spread of the network from individual nodes. The colour schemes are coded by thematic area and web/link strength between the keywords. For example, the adult male node is the largest node located close to the middle of the diagram, indicating that adult male firefighters are the most frequently studied key terms in firefighters. Nodes located on the periphery of the diagram are the least occurring keywords, with the lowest network strength to other nodes/co-occurrences.

### 2.3. Inclusion and Exclusion Criteria

The inclusion criteria were studies involving all types of firefighters, that used CVD risk factors and/or musculoskeletal health/disorders/injuries and/or physical fitness and/or occupational/professional/work/job performance (Table 2). Studies involving all types of firefighters, active duty, seasonal, contract, volunteer, new recruits, of all ages, genders, and ethnicities were included. Studies that did not meet the purpose of the literature review (e.g., not using two or more of the variables, i.e., CVD risk factors, musculoskeletal health, physical fitness, or occupational performance) were excluded. In addition, intervention and review studies were excluded from this review. To limit the possibility of selection or reviewer bias, all studies related to the present review were included.

Key terms were searched in various combinations in PubMed, Web of Science, and Scopus (Table 3). In total, 807 articles were found in PubMed, 973 in Web of Science, and 823 in SCOPUS, totalling 2603 articles. Four studies were found from grey literature searchers. After each search, the search results were exported as either txt, RIS or BibTeX files, and files were then imported into Zotero™ reference manager, for further screening and checking for duplications.

### 2.4. Screening Procedure

In total, 2603 articles were identified through electronic database searches and four articles through a search of the grey literature (Figure 2). After removal of the duplicates (Zotero™), 1188 articles remained, which were then screened for eligibility using the titles and abstracts, and 980 articles were excluded for not meeting the review requirements (title, abstract, and keywords). The remaining 209 articles were screened based on the inclusion and exclusion criteria, as well as the full-text, where 161 articles were excluded for the following reasons: being an intervention study; the relationship between the variables not clearly described; inconclusive results reported; the outcome variables were not aligned with the scope of this review. A total of 46 articles were finally identified, which were included in the narrative review.

### 2.5. Data Extraction

The principal investigator designed a spreadsheet in Microsoft Excel® for the data extraction. The extraction of data is a descriptive summary of the results that align with the objectives of the current review [38]. Five categories of data were extracted from each article and were populated in the spreadsheet. The categories included reference (author), year, sample size, research design, and outcomes of the study. Data were extracted by the authors JR and LL.

## 3. Results

From the 46 studies, 26 were published from North America (USA = 21; Canada = 5), 10 studies were published from Europe (Central Europe = 8; United Kingdom = 2), 3 studies were published from Asia (1 = Korea; 1 = Tehran; 1 = China), 2 were published from Australia, and 1 study from Africa (Ghana). In the literature, most studies investigated the relationship between CVD risk factors and physical fitness or the relationship between physical fitness and occupational performance. The high morbidity and mortality rates seen in firefighters reflected the relatively high volume of literature in these areas, as over 45% of firefighter fatalities were due to poor or deleterious cardiovascular health [15].

The effects of musculoskeletal health have been understudied in firefighters, particularly in relation to CVD risk status and occupational performance [39, 40]. These factors, ultimately, result in impaired occupational performance in firefighters, placing them at significant risk of CVD and musculoskeletal injury [15, 39]. The following results are separated into themes concerning the relationships between the variables.

### 3.1. Cardiovascular Disease Risk Factors and Musculoskeletal Health

Six studies investigated the relationship between cardiovascular and musculoskeletal health. The results of the studies are summarized in Table 4. The results indicated that age, obesity, and cigarette smoking were significantly associated with reduced musculoskeletal health, specifically, in the lower back and lower extremities [19, 21, 22].

Negm et al. [45] conducted a cross-sectional study on 294 full-time male firefighters in Hamilton Trenholm, Canada, investigating their musculoskeletal health. The study reported that aged firefighters (≥42) were significantly related to poorer musculoskeletal health, specifically to lower extremity disability (*p* = 0.03) and severe low back pain (*p* < 0.001). In addition, aged firefighters were more likely to have multiple sites with poor or severe musculoskeletal health. Similarly, Jang et al. [43] conducted a study on 392 full-time firefighters in Dongguk, Goyang, Korea, and found that age was a significant predictor of lumbar intervertebral disc degeneration (*p* < 0.05) in firefighters. This was supported in another study, which reported that age was a significant predictor of back pain (*p* = 0.002) in firefighters [44]. Likewise, an earlier study by Gordon and Lariviere [42] on 252 full-time male and female firefighters from Ontario, Canada, reported that age was a significant predictor of musculoskeletal injury (OR = 6.49, *p* < 0.05). Aged firefighters are more likely to have poor musculoskeletal health compared to their younger counterparts. [42].

Damrongsak et al. [44] conveniently sampled 298 male firefighters in the South-eastern regions of the United States (US). The study investigated the predictors of back pain and reported that the combination of occupational stress, age, history of back pain, and obesity (BMI) were significant predictors of current back pain in firefighters (*χ*^2^ = 127.84, df = 4, *p* < 0.0001). Jahnke et al. [22] conducted a cross-sectional study on 347 full-time firefighters from Kansas, Missouri, Iowa, Nebraska, North Dakota, South Dakota, Colorado, and Wyoming which investigated the factors that affected injury prevalence. The study noted that obesity (BMI and WC) was significantly related to poor musculoskeletal health, and increased the risk of firefighters sustaining acute musculoskeletal injuries when on duty by 5.2 and 2.8 times, respectively. In addition, another study reported that cigarette smoking was significantly related to musculoskeletal injuries in firefighters [21]. Similarly, Poston et al. [41] reported that, in 478 full-time male firefighters age, obesity and smoking status were significant predictors of poor musculoskeletal health (*p* < 0.001). Moreover, firefighters categorised with class II and III obesity were more likely to sustain injuries (OR = 4.89). Likewise, Jahnke et al. [21] reported that firefighters who were former smokers were more likely to sustain a musculoskeletal injury compared to nonsmokers (OR = 1.84).

### 3.2. Cardiovascular Disease Risk Factors and Physical Fitness

Fourteen studies investigated the relationship between CVD risk factors and physical fitness in firefighters. The results of the studies are summarized in Table 4. Overall, higher levels of physical fitness, particularly cardiorespiratory fitness, were related to improved CVD risk status in firefighters [8, 29, 46–48, 78]. This relationship has been studied, more thoroughly in firefighters, as both factors represent essential components in firefighters' health, wellness, and occupational performance [8, 47].

Kiss et al. [51] investigated cardiorespiratory fitness in 1225 firefighters from East-Flanders Province, Belgium. The study reported that age (*R*^2^ = 0.28, *p* < 0.001) and obesity (*R*^2^ = 0.28, *p* < 0.001) were significant predictors of cardiorespiratory fitness (Table 4). The study noted that age and obesity should be monitored closely in firefighters, especially between the ages of 30–50 years, when the risk escalates exponentially. A limitation of the study was that only male firefighters were included, due to the low number of female firefighters. Kirlin et al. [54] investigated the effect of age on physical fitness in a sample of 97 female firefighters from San Diego, USA. The study reported that, in female firefighters, age was significantly related to cardiorespiratory fitness (*p* < 0.001). Interestingly, age was not associated with muscular endurance in females.

Phillips et al. [7] investigated the effect of obesity on physical fitness in 414 full-time male firefighters from Alberta, Canada. The study found that obese firefighters had a significantly shorter treadmill time (*p* < 0.05) and lower cardiorespiratory fitness (*p* < 0.05) compared to firefighters with normal body weight. A study that investigated the CVD risk factors in 294 full-time firefighters in Colorado, USA, reported that improved cardiorespiratory fitness was a significant predictor of better cardiovascular risk status (OR = 2.87, *p* < 0.05) [55]. This was supported by another study which reported that increased cardiorespiratory fitness was inversely related to deleterious cardiovascular risk status (*p* < 0.001) in male firefighters [46]. Barry et al. [56] investigated the relationship between body composition and physical activity on cardiorespiratory fitness in 29 conveniently sampled full-time male firefighters and found that central obesity (*β* = 0.482, *p* < 0.001) and vigorous physical activity (*β* = 0.560, *p* < 0.001) were significant predictors of cardiorespiratory fitness. However, the small sample size limited the generalizability of the results. The results of Barry et al. were supported by an earlier study by Punakallio et al. [24] which found that firefighters who exercised at least four to five times a week (*p*=0.016) maintained cardiorespiratory fitness throughout their careers, and that aging (*p*=0.048), regular smoking (*p*=0.048), and alcohol consumption (*p*=0.018) were significant predictors of a decline in cardiorespiratory fitness.

Baur et al. [47] conducted a large-scale cross-sectional study on 968 male firefighters from the US and reported that higher cardiorespiratory fitness was significantly associated with improved CVD risk status, specifically, to lower systolic blood pressure (SBP) (*p* < 0.001), body fat percentage (BF%) (*p* < 0.001), triglycerides (*p* < 0.001), low-density lipoprotein cholesterol (LDL-C) (*p* < 0.001) total cholesterol (TC) (*p*=0.005), and total/high-density lipoprotein cholesterol ratio (TC/HDL-C) (*p* < 0.001). Higher cardiorespiratory fitness was also associated with higher HDL-C [47]. Similarly, Seyedmehdi et al. [29], in 157 full-time male firefighters in Tehran, reported that cardiorespiratory fitness was significantly correlated with age (OR = 4.86, *p*=0.011), obesity (BM and WC) (OR = 4.69, *p*=0.009), cigarette smoking (OR = 6.64, *p*=0.045), physical inactivity (OR = 5.53, *p*=0.003), blood cholesterol (OR = 5.44, *p*=0.010), SBP (OR = 7.50, *p*=0.045) and diastolic blood pressure (DBP) (OR = 2.70, *p*=0.045), and heart rate (*p*=0.001). Strauss et al. [8] also studied about 97 full-time firefighters in Germany and reported that age (*β* = −2.04, *p* < 0.001), obesity (BMI, WC, and BF%) (*β* = −1.07; *β* = −3.23; *β* = −2.20, *p* < 0.001), SBP (*β* = −1.58, *r* = 0.007), DBP (*β* = −1.36, *p*=0.001), triglycerides (*β* = −12.38, *p*=0.0024), and total cholesterol (*β* = −4.90, *p*=0.0067) were significant predictors of cardiorespiratory fitness. Likewise, Espinoza et al. [57] investigated 76 volunteer Chilean male firefighters and reported that obesity (*β* = −10.8, *p* < 0.001), central obesity (*β* = −7.71, OR = 12.35, *p* < 0.001), and altered glucose (*β* = −4.4, OR = 2.87, *p*=0.019) were significant predictors of cardiorespiratory fitness. The study also found that age (*r* = −0.36, *p* < 0.001), heart rate (*r* = −0.27, *p* < 0.01), SBP (*r* = −0.24, *p* < 0.03), and DBP (*r* = −0.25, *p* < 0.02) were negatively correlated with cardiorespiratory fitness. [57] The previous studies only investigated male firefighters, which limits the generalizability of the results.

Yang et al. [59] investigated the association between muscular endurance (push-up capacity) and CVD risk factors in 1562 full-time firefighters in Indiana, USA, and found that push-up capacity was significantly related to CVD risk factors, specifically, age (*p* < 0.001), obesity (*p* < 0.001), blood pressure (BP) (*p* < 0.001), TC (*p*=0.02), LDL-C (*p*=0.04), triglycerides (*p* < 0.001), blood glucose (*p* < 0.001), and smoking (*p* < 0.001). A limitation of the study was that the researchers investigated push-ups only and did not control for other physical fitness measures, which could have influenced the results. Also, the result cannot be generalized to women or older firefighters, as the cohort consisted of middle-aged male firefighters only. Another study on the impact of obesity on back and abdominal muscular endurance in 83 full-time firefighters from Florida, USA, 57 reported that back and core muscular endurance was 27% lower for obese firefighters compared to nonobese firefighters, and that significant negative correlations were reported between back endurance and age (*r* = −0.22, *p* < 0.05) and obesity (*r* = −0.44, *p* < 0.01) and between core endurance and obesity (*r* = −0.47, *p* < 0.01). Studies by Poplin et al. [50, 53] reported similar results in which aging was negatively correlated with V̇O_2max_ (*r* = −0.368, *p* < 0.05), and flexibility (*r* = −0.160, *p* < 0.05), and that BF% was negatively correlated with V̇O_2max_ (*r* = −0.448, *p* < 0.05), grip strength (*r* = −0.191, *p* < 0.05), and flexibility (*r* = −0.135, *p* < 0.05).

Baur et al. [48] investigated the relationship between physical fitness and autonomic abnormalities (heart rate recovery, chronotropic insufficiencies, ST elevation or depression, ventricular tachycardia, sustained supraventricular tachycardia, and exercise-induced left or right bundle branch block) in 1149 full-time male firefighters from the USA and reported that cardiorespiratory fitness was inversely associated with ECG and autonomic abnormalities (OR = 0.63, *p* < 0.001), and remained significant after being adjusted for age (*p* < 0.001), BMI (*p* < 0.001), and metabolic syndrome (*p* < 0.001). Similarly, Porto et al. [58] reported that a positive correlation existed between higher cardiorespiratory fitness and overall cardiac autonomic function and parasympathetic activity (*p* < 0.001). Autonomic function provides a valuable measure in determining CVD risk in firefighters and requires more research to investigate its use.

### 3.3. Cardiovascular Disease Risk Factors and Occupational Performance

Six studies examined the relationship between CVD risk factors and occupational performance in firefighters. The results of the studies are shown in Table 4. Walker et al. [52], in 73 full-time male Australian firefighters, found significant differences between age-groups for cardiorespiratory fitness (*ω*^2^ = 0.23, *p* < 0.001), overall strength (*ω*^2^ = 0.21, *p*=0.001), dummy drag (*ω*^2^ = 0.26, *p* < 0.001), and hose drag (*ω*^2^ = 0.46, *p* < 0.001). Similarly, Nazari et al. [26] reported that age was a significant predictor of hose drag (*β* = 0.48, *p*=0.003) and stair climb (*β* = 0.46, *p*=0.030) in firefighters. Saari et al. [62] investigated the influence of age on occupational performance in 74 full-time male firefighters in Kentucky, USA, reported that aging correlated with occupational course time (*r* = 0.297, *p*=0.017). Aged firefighters (≥37 years) had an 8.8% longer completion time compared to younger firefighters. The study also reported a trend between obesity and course time, but the relationship was not statistically significant. Another study found that aging (*r* = 0.42, *p* < 0.01) and obesity (*r* = 0.57, *p* < 0.01) were significantly correlated with poorer performance in the physical ability test (PAT) in firefighters [73]. In addition, a high resting heart rate as correlated with poorer occupational performance (*r* = 0.36, *p* < 0.01). These results were supported by two studies which reported that high BF% was associated with poor performance in the physical ability tests [63], and that aging and fat mass were significant predictors of work inefficiency in firefighters [64].

Firoozeh et al. [61] conducted a study on 375 full-time male Australian firefighters and reported that age (*r* = −0.277, *p*=0.001) and obesity (*r* = −0.187, *p*=0.001) were negatively correlated with work ability, and that leisure-time physical activity (LTPA) (*r* = 0.206, *p*=0.001) correlated to work ability. Similarly, an earlier study by Airila et al. [60] reported that, in 403 male Finnish firefighters, age (*r* = −0.33, *p* < 0.01), obesity (*r* = −0.15, *p* < 0.01), and cigarette smoking (*r* = 0.10, *p* < 0.05) were negatively correlated with work ability, and that physical exercise (*r* = −0.15, *p* < 0.01) correlated with work ability and work demands. A model reported that various CVD risk factors, such as alcohol consumption, obesity, cigarette smoking, and physical activity were significant predictors of work ability (*R*^2^ = 0.48, *p* < 0.001) [60]. Nazari et al. [39] reported that aged firefighters (≥45 years) experienced significantly more physical work limitations than their younger counterparts (*β* = 0.27, *p*=0.004). In the studies by Firoozah et al., Airila et al., and Nazari et al., work ability was self-reported, and not verified using simulation tasks, which could include subjective bias in the reporting.

In contrast to the previous studies, Phillips et al. [7] reported that obese firefighters had significantly faster completion times for the hose drag (*r* = −0.44, *p* < 0.05), weighted-sled pull (*r* = −0.36, *p* < 0.05), forcible entry (*r* = -0.27, *p* < 0.05), and victim rescue (*r* = −0.21, *p* < 0.05), whereas normal weight firefighters only performed better on the ladder climb task (*r* = −0.24, *p* < 0.05). However, the uniformity of body mass across participants was not controlled, and the results may not be a true reflection of the effect of obesity on occupational performance.

### 3.4. Musculoskeletal Health and Physical Fitness

Five studies investigated the relationship between musculoskeletal health and physical fitness in firefighters. The results are summarized in Table 4. All aspects of physical fitness play an important role in the maintenance of musculoskeletal health, through increased skeletal muscle strength, connective tissue integrity, and increased bone mineral density [45, 79–81]. High levels of physical fitness may prove beneficial for firefighters and can significantly reduce the incidence of injuries [79].

Butler et al. [66] reported that three flexibility movements (fundamental movements) were significant predictors of injuries in firefighters, namely, the sit-and-reach (*β* = 0.218, *p* < 0.05), push-up (*β* = 0.190, *p* < 0.05), and deep squat (*β* = 0.266, *p* < 0.05). Firefighters who performed poorly on the sit-and-reach, deep squat, and push-up were 1.21, 1.24, and 1.30 times more likely to sustain injury, respectively [66]. Flexibility, particularly related to fundamental movements, may prove to be an important measure in preventing injuries in firefighters.

Wynn and Hawdon [65] conducted a study in 398 full-time and 48 part-time recruits with no fitness standard, and 198 full-time and 206 part time recruits where a minimum cardiorespiratory fitness standard of 42 mL·kg·min was applied, and reported that poor musculoskeletal health was more likely to occur in the service where no physical fitness standard was required. In addition, higher cardiorespiratory fitness was a significant predictor of lower incidence of musculoskeletal health issues [65]. A similar result was reported by Poplin et al. [50] where a longitudinal study was conducted investigating the effect of cardiorespiratory fitness on musculoskeletal health in 577 full-time firefighters in the Southwestern States, USA. The results indicated that firefighters in the lowest fitness categories were 2.2 times more likely to sustain injuries, compared to those in the highest fitness categories. Furthermore, the study found that firefighters with a cardiorespiratory fitness between 43 and 48 mL·kg^−1^·minute^−1^ were 1.38 times more likely to sustain injury. Improving cardiorespiratory fitness by one metabolic equivalent was shown to reduce the risk of any injury by 14%. A later study by Poplin et al. [53] reported a similar result with 799 full-time firefighters which noted that firefighters with lower cardiorespiratory fitness were 1.82 times more likely to sustain injury. When injury types were restricted to sprains and strains exclusively, firefighters with lower cardiorespiratory fitness were 2.90 times more likely sustain an injury [53].

In contrast to the previous studies, a study by Damrongsak et al. [44] found that high physical fitness did not reduce the incidence of back pain in firefighters. Similarly, Gordon and Lariviere [42] noted that higher cardiorespiratory fitness was not significantly associated with better musculoskeletal health in firefighters. Butler et al. [66] also reported a similar result, where cardiorespiratory fitness was not a predictor of injuries in firefighters. Interestingly, a study by Jahnke et al. [21] in 462 full-time firefighters reported that firefighters who exercised regularly while on duty were 4.6 times more likely to sustain an exercise-related injury. In addition, higher levels of cardiorespiratory fitness and muscular strength increased exercise-related musculoskeletal injury risk by 1.06 and 4.03 times, respectively, while on-duty. However, regular exercise when on duty did reduce the incidence of injuries outside of the workplace. High workload when on duty, compounded by exercise or training workload and inadequate recovery possibly produced a burdensome triad that reduced musculoskeletal health and contributed to the increased incidence of duty-related injury [78, 82].

### 3.5. Musculoskeletal Health and Occupational Performance

Five studies investigated the relationship between musculoskeletal health and occupational performance in firefighters. The results of the studies are indicated in Table 4. Firefighting is a physically demanding occupation that requires the musculoskeletal system to be in good condition for firefighters to perform at peak performance [17, 39, 45, 83]. Chronic musculoskeletal pain and chronic disorders negatively affect performance and reduce endurance capacity and force production [79]. Musculoskeletal health is essential for satisfactory work performance in any emergency occupation, particularly in firefighting [80, 83].

Punakallio et al. [67] investigated the effect of musculoskeletal health on self-reported work ability in 411 male firefighters from Helsinki Finland and reported that musculoskeletal pain (MSP) in more than one site was at increased risk of diminished work ability. The study also found that musculoskeletal health isolated to the low back (OR = 1.9), forearm, and hand (OR = 1.9) predicted diminished work ability. In addition, firefighters who were on disability pension reported having poor work ability and more musculoskeletal health concerns at baseline. Furthermore, firefighters engaging in average-to-high physical workload when on duty was a significant risk factor for retiring due to deteriorated musculoskeletal health (OR: 3.1 to OR: 5.3, respectively). Similarly, Saremi et al. [69] in 250 Tehran firefighters reported an inverse relationship between work-ability index and musculoskeletal discomfort in the wrists (*p* = 0.007, *r* = –0.170), legs (*p* = 0.042, *r* = –0.129), and ankles (*p* = 0.005, *r* = –0.176). Kodom–Wiredu [68] examined 320 full-time firefighters in the Greater Accra region of Ghana found that work-related musculoskeletal disorders (WRMSD) were significantly related to work demands (*r* = 0.03) and task characteristics (*r* = 0.26), and that increased work demands (*β* = 0.226, *p* < 0.01) and task characteristics (*β* = 0.214, *p* < 0.01) were significant predictors of WRMSDs. Similarly, Nazari et al. [39] in 325 full-time Canadian firefighters found a significant relationship between musculoskeletal health and self-reported physical work limitations. The study noted that firefighters with spinal pain (*p* = 0.01) experienced significantly limited occupational output. In addition, the number of musculoskeletal pain sites (*p* = 0.02) were significant predictors of limited occupational output and work performance [39]. MacDermid et al. [40] in the sample of 293 full-time Canadian firefighters reported that firefighters with moderate-to-severe muscle and joint complaints took on average 10 seconds longer to complete functional performance tasks, but the results were not statistically significant [40]. However, the majority of studies were self-reported measures for work ability and, therefore, may be subject to reporting bias. More research needs to be conducted in this particular area, where firefighters with pain or deteriorating musculoskeletal health are assessed while performing simulated tasks, that would be faced while on active duty.

### 3.6. Physical Fitness and Occupational Performance

Ten studies investigated the relationship between physical fitness and occupational health in firefighters. The results are summarized in Table 4. Due to the inherently physical nature of firefighting, physical fitness is regarded as a fundamental component for optimum occupational performance. Various studies showed that muscular strength, muscular endurance, and cardiorespiratory fitness were significantly related to firefighter occupational ability and performance [83, 84].

von Heimburg et al. [70] in 13 male Norwegian firefighters reported that cardiorespiratory fitness was a significant predictor of simulation performance times (*r* = 0.53, *p*=0.05). Furthermore, stronger, heavier, and taller firefighters had a significantly lower performance time (*p*=0.01). The authors noted that the small sample size of the study negatively impacted the generalizability of the results. Another study with 20 male firefighters reported a moderately strong and inverse relationship between cardiorespiratory fitness and performance time in firefighter simulation protocols [84]. The small sample size and using male firefighters only limits the generalizability of the results. Skinner et al. [77] examined the predictors of task performance in 42 male aerial firefighters from Queensland Australia and found that cardiorespiratory fitness and body composition were inversely correlated to firefighting simulation protocol performance time. Poor body composition was significantly related to slower performance time on the simulation. Similarly, Xu et al. [63] reported that poor body composition (higher BF%) was associated with poor performance on the work ability test in 20 full-time Chinese firefighters. Superior cardiorespiratory fitness, and upper and lower body muscular power, was inversely related to the completion times in the work ability test.

Sheaff et al. [72] in 33 firefighters reported that certain physical fitness parameters, such as cardiorespiratory fitness (*r* = 0.602, *p* < 0.001), upper body strength (*r* = 0.485, *p* < 0.001), and grip strength (*r* = 0.504, *p* = 0.009), were significantly related to performance times in the Candidate Physical Ability Test (CPAT). Cardiorespiratory fitness was a significant predictor of CPAT performance. Similarly, Michaelides et al. [73] reported that firefighter ability test completion times were significantly related to abdominal strength, relative power, upper-body muscular endurance, and upper body strength. The study also noted that poor performance on the ability test was associated with poor body composition. However, the studies by Sheaff et al. and Michaelides et al. used small sample sizes with few females, which negatively impacted the statistical power and generalizability of the results. Nazari et al. [26] noted that right-hand grip strength was a significant predictor of hose drag times, and that lower body strength was a significant predictor of stair climb in firefighters. In addition, cardiorespiratory fitness was significantly correlated with the task times for the hose drag (*r* = −0.30, *p* = 0.01) and stair climb (*r* = 0.31, *p* = 0.01), and that increased lower body strength was significantly correlated with hose drag time (*r* = −0.20, *p* = 0.01) [26]. The importance of muscular strength in occupational performance was emphasized by Kleinberg et al. [75] who reported that lower body strength (*r* = 0.560, *p* < 0.001) was significantly associated with stair climb time in firefighters that remained significant after adjustment for age and BMI.

A later study by Heimburg et al. [74] in 63 full-time Norwegian firefighters reported that the treadmill and push up tests (*r* = −0.42, *p* < 0.001), squat and raise (*r* = −0.54, *p* < 0.001), and horizontal chest to bar pullups (*r* = −0.34, *p*=0.1) were significantly related to faster simulation task times. Firefighters had a higher cardiorespiratory fitness and were stronger completed the simulation protocol faster (*p* < 0.05). Anomalies in the results existed, where firefighters with below average strength completed the test the quickest, indicating that a minimal strength was needed to perform well, and strength beyond that point did not improve performance times [74]. Comparably, a study on 68 full-time English firefighters from the United Kingdom reported that cardiorespiratory fitness was the strongest predictor of firefighter simulation task time [76]. However, contrary to the previous studies, muscular strength was not found to be a significant predictor of firefighter simulation task time [76].

## 4. Discussion

In the present review, the most frequent relationships investigated were between CVD risk factors and physical fitness (fourteen studies) and between physical fitness and occupational performance (ten studies). This may be due to CVD risk factors and physical fitness being especially important for firefighters' career longevity and work performance [2, 3, 15]. In addition, the relationships between CVD risk factors, musculoskeletal health, and between musculoskeletal health and physical fitness were understudied, especially in relation to occupational performance. However, studies investigating musculoskeletal health and occupational performance reported that musculoskeletal health negatively affected firefighter performance.

There was a significant inverse relationship between increased CVD risk factors and reduced musculoskeletal health in firefighters, which was particularly related to increased age, obesity, cigarette smoking, and physical inactivity. [22, 24, 43–45] Aging caused a decrease in bone mineral density, a decrease in ligament and tendon elasticity, and reduced tissue recovery and healing time that predisposed firefighters to injury while on duty [35, 45]. Obesity increased the overall force placed on the musculoskeletal system, particularly when engaged in activities of vigorous-intensity, such as firefighting [12, 85, 86]. As seen in Figure 3, obese firefighters fatigue at a faster rate, resulting in acute traumatic injuries and chronic overuse injuries [22]. Fatigue causes inadequate energy absorption, as well as reduced control and regulation of limb movements [87]. The present review shows that smoking has a negative effect on tendon health, bone mineral density, and hormone regulation, particularly oestrogen and cortisol [34], and may partially explain the decreased musculoskeletal health and increased injury risk in firefighters. Physical activity has a protective effect on the musculoskeletal system, particularly vigorous-intensity activity [88]. Unfortunately, research shows that firefighters tended to be physically inactive, with many not reaching the minimum weekly recommended amount of physical activity [9, 27, 47, 56, 78]. Aging, obesity, cigarette smoking, and physical inactivity negatively affected both cardiovascular and musculoskeletal health (Figure 3), and should be identified early in firefighters and given particular attention in the latter stages of their careers.

Cardiovascular disease risk factors, such as age, obesity, lipid profile, blood glucose, blood pressure, cigarette smoking, and physical inactivity were shown to be significantly related to cardiorespiratory fitness and muscular endurance in firefighters [9, 27, 29, 47, 48, 51, 54, 56, 58, 59]. In addition, back and core endurance were significantly related to age and obesity in firefighters [49]. Furthermore, CVD risk factors were significantly related to cardiorespiratory fitness in firefighters [46, 55]. The progressive deterioration in cardiovascular, pulmonary, and musculoskeletal health with increasing age accounted for the decrease in cardiorespiratory fitness and muscular endurance in firefighters [27, 89]. This is further exacerbated by the constant chemical and fume inhalation, which negatively effects pulmonary functioning in firefighters [90]. In the case of obesity, the increased weight and peripheral resistance to blood flow increased the stress and workload placed on the musculoskeletal and cardiovascular systems, resulting in a decrease in endurance capacity [22, 91]. Consequently, with aging, this effect is further compounded by the biological deterioration in cardiovascular, musculoskeletal, and pulmonary health [89].

An altered lipid profile negatively affected cardiorespiratory fitness in firefighters [9, 29, 47]. This relationship can be explained in a study conducted by Rumora et al. [92], where the results showed that dyslipidaemia caused altered mitochondrial functioning that decreased energy production. Reduced mitochondrial function negatively affects aerobic performance [93]. High blood glucose concentrations negatively affects glucose homeostasis and glucose metabolism, and together with altered mitochondrial function in skeletal muscles, these negatively affect endurance capacity [94]. Elevated DBP and SBP also negatively affect cardiorespiratory capacity, due to altered diastolic atrial and ventricular filling, subsequently reducing the stroke volume of the heart. In addition, the increase in blood pressure increases the cardiac afterload, further reducing stroke volume and cardiac output (Figure 3) [95]. Cigarette smoking causes pulmonary damage and reduces the oxygen-carrying capacity in the blood that may explain the inverse relationship seen between the two factors [34]. Physical inactivity augments the progressive decline in the cardiovascular, pulmonary, and musculoskeletal systems and, thereby, partially explains the linear relationship with cardiorespiratory fitness [48, 96].

Aging, obesity, cigarette smoking, and physical inactivity were the CVD risk factors related to poor physical fitness, occupational performance, and work ability in firefighters [26, 52, 60–62, 69, 73]. In addition, increased leisure time physical activity was positively related to work ability in firefighters [61]. Firefighting often requires firefighters to perform complex, vigorous-intensity activities that strain all systems of the body. Aging generally reduces muscular force production, cardiorespiratory efficiency, tissue elasticity, healing, and repair, more especially when combined with an unhealthy lifestyle [89]. This directly affects the performance of occupational tasks and partially explains the reduction in work performance with progressively advancing age [27, 62]. The pervasive physical inactivity and unhealthy lifestyle that often accompanies firefighters as they age further exacerbates the deleterious effects of aging [9, 56, 78]. In addition, obesity places significant strain on all bodily systems, causing premature fatigue and, consequently, reduced occupational performance [73]. As a result of cigarette smoking, the reduction in pulmonary capacity and oxygen-carrying capacity also adversely affects occupational performance [27, 96].

One study reported that increased body mass of firefighters related to better performance on certain firefighter specific tasks, especially tasks requiring significant muscular [7]. The relationship between increased body weight and a reduction in task completion times may be related to the increase in muscle mass that accounted for the increase in body mass rather than an increase in fat [7]. Muscle strength can be a significant factor in the optimal performance of firefighters. Heavier firefighters may perform better on strength-based occupational tasks but perform worse on cardiorespiratory fitness tests [7, 26, 29, 47, 97]. Consequently, for optimal work performance, firefighters require delicate balance between cardiovascular fitness and muscular strength for occupational task performance.

Current literature indicated that increased cardiorespiratory fitness was significantly related to fewer musculoskeletal injuries in firefighters, and that three fundamental movements related to flexibility could predict injuries, i.e., the sit-and-reach, push-up, and deep squat [50, 53, 65]. Any form of physical activity has a protective effect on musculoskeletal health, whether aerobic or anaerobic in nature and, furthermore, performing regular aerobic exercise translates into improved cardiorespiratory fitness [9, 21]. Flexibility, particularly in the lower back, hamstrings, and hips, is related to reduced injury incidence [66]. Functional flexibility is a critical fitness parameter in firefighters, as their work requires awkward movement patterns, such as bending, lifting, and crawling [66, 98].

In contrast, one study reported that firefighters who exercised were not at lower risk of sustaining musculoskeletal injury [44]. Another study found that firefighters who exercised, while on duty, were at higher risk for sustaining work-related injury [21]. A possible reason for the increase in injury incidence in firefighters who exercised while on-duty may be due to the chronic overload placed on the muscular system, which led to acute overload injuries [19, 99]. Firefighters who participate in regular physical activity should monitor their overall workload and balance the workload with adequate recovery time in order to reduce the incidence of injury. Finding this “sweet spot” may prove essential to maintaining optimal musculoskeletal health and preventing injury.

Poor musculoskeletal health negatively affected occupational performance and work ability in firefighters, and was particularly related to low back, forearm, wrist, hand, and leg discomfort [67–69]. Increased work demands and the various types of task performed were significantly related to musculoskeletal disorders [68]. Spinal pain and multiple injuries were significantly related to limitations in occupational output and work performance [39]. Firefighters with moderate-to-severe muscle and joint problems took 10 seconds longer to complete occupational performance tasks [40]. Injuries and chronic pain reduced muscular force production, and altered movement patterns to compensate for the workload on the injured or painful area [39]. The reduced force production and protective movement patterns acted as a subconscious protective mechanism that may negatively affect on-duty performance [39, 80, 100]. These altered movement patterns may become particularly apparent in emergency situations, which require maximum force production, muscular endurance, and coordination, such as door breaches, equipment carries, and hose drags. However, more research is needed on the extent to which the location and severity of injuries negatively affected occupational performance, especially in firefighter specific tasks.

Cardiorespiratory fitness was significantly related to all components of occupational task performance in firefighters [26, 63, 72, 73, 77, 84, 101]. In addition, upper body muscular strength and endurance were significant predictors of occupational performance [26, 72, 73]. Quadriceps strength was a significant predictor of stair climb performance in firefighters [75]. Firefighters routinely have to perform activities that are exhaustive on the upper body, such as door breaches, hose carries, hose drags, victim drags, and victim carries [74, 76, 102]. In addition, firefighting simulation tasks require predominantly upper body strength and endurance [63, 70, 74, 76, 77]. Therefore, firefighters with greater upper body strength and endurance generally perform better on these tasks increased fat mass and lower lean mass were significantly related to poor occupational performance [63, 77]. Poor performance in firefighters with unhealthy body composition may be related to the increased muscular workload, as a result of the increased adiposity and lower proportion of lean body mass [6, 7, 26, 63, 76, 77].

In firefighting, all health-related physical fitness parameters positively affected occupational performance [70, 74]. However, beyond the threshold of desirable physical fitness, this point further improves in fitness that had little benefit on occupational performance [74]. This indicated that firefighters may be competent in performing the occupational tasks, due to having sufficient physical fitness, despite having underlying cardiovascular and musculoskeletal health challenges. Consequently, firefighters may be on active duty, while having underlying health concerns, which may account for the high cardiovascular-related morbidity and mortality [2, 11, 15, 103], and the high rate of musculoskeletal related complaints that resulted in early retirement in this population [19, 20, 69, 81]. All aspects of the firefighters' health should be thoroughly monitored throughout the firefighters' career to ensure career longevity and decrease the incidence of duty related-deaths and early retirement. As previously discussed, larger and heavier firefighters, who are often obese, tended to perform better on strength-based tasks, such as the door breach, equipment carry, and victim drags, but performed worse on the cardiorespiratory fitness tests, such as the stair climb and ladder raise tests, due to their excess body weight that acted as a hindrance in these tasks [6, 26, 74, 76]. While overweight and obese firefighters may pass the simulation protocols, they remain at increased risk for early retirement, morbidity, and mortality.

As seen in Figure 3, CVD risk factors, musculoskeletal health, and physical fitness play a significant role in firefighter occupational performance. Increased CVD risk increases the cardiovascular strain associated with firefighting and, in the same vein, reduced musculoskeletal health, increased musculoskeletal pain and the risk of musculoskeletal disorders, thereby, reducing muscular force and occupational. Poor physical fitness increases the cardiovascular strain and reduces musculoskeletal health that causes an overall decrease in cardiorespiratory capacity and musculoskeletal strength, endurance, and flexibility, which is further compounded by poor body composition. Together, these factors cause increased fatigue and reduced the occupational performance for any given task and, as a consequence, leads to slower task completion times and poor overall occupational performance in firefighters.

The literature indicates that most CVD risk factors have a negative effect on physical fitness [9, 27, 29, 47, 48, 51, 54, 56, 58, 59], and that physical fitness and musculoskeletal health are significantly related [50, 53, 65]. Because physical fitness is related to occupational performance, the assumption can be made that increased CVD risk factors and reduced musculoskeletal health would result in reduced occupational performance in firefighters. However, this needs to be investigated further.

### 4.1. Strengths of the Study

The majority of studies were conducted in the USA, with relatively small sample sizes, and involved males primarily, thus limiting the generalizability of the results to the broader firefighting population. The narrative review involved an iterative process of checking and cross-checking in order to ensure a narrative review of the highest quality and rigour. The quality assessment process started with the identification of the search terms and constructing the search string that was database specific, and ended with the data extraction and interpretation of the findings.

### 4.2. Limitations of the Study

The limited number of electronic databases searched and that only articles in English and in full-text were considered for selection are limitations to the current literature review. There were no qualitative studies included in the current study and, therefore, only quantitative studies were used. No critical appraisal or risk of bias tools were used to grade the included studies, however, the authors attempted to maintain methodological transparency and rigor throughout the review process.

## 5. Conclusion

Cardiovascular disease risk factors and physical fitness were the most frequently studied areas in firefighters and were significantly related. Cardiovascular disease risk factors were significantly related to cardiorespiratory fitness in firefighters, particularly age, obesity hypertension, dyslipidaemia, cigarette smoking, and physical inactivity. In addition, physical fitness, especially cardiorespiratory fitness, was found to be significantly related to overall occupational performance. Certain CVD risk factors were significantly related to musculoskeletal health, and in particular, obesity and cigarette smoking. Cardiovascular risk factors, such as obesity and age were significantly related to worse occupational performance. Musculoskeletal health, in relation to occupational performance, is understudied; however, the results indicated that poor musculoskeletal health was related to work and performance limitations. Overall, the research indicated that aged, obese, and unfit firefighters who smoked cigarettes and were physically inactive were at the highest risk for CVD and musculoskeletal health complications, and produced unsatisfactory occupational performance. Moreover, most CVD risk factors were related to low levels of physical fitness. Due to limited research, significant gaps still remain in the literature and, in particular, regarding the relationship between musculoskeletal health and occupational performance. In addition, firefighters are understudied in developing countries, and, in particular, African countries.

### 5.1. Recommendations

More research should be conducted investigating the relationship between CVD risk factors and occupational performance, between musculoskeletal health and physical fitness, and between musculoskeletal health and occupational performance. In addition, females were underrepresented in many of the studies and, therefore, more research involving female firefighters should be conducted. The majority of studies on firefighters were conducted in developed countries and the results cannot be generalized to firefighters in developing countries. Consequently, more research is needed in developing countries to provide a more holistic view of firefighters globally. This will inform policy makers, as well as fire departments on the most significant factors influencing occupational performance in both developed and developing countries. There is a need by the fire services to implement corrective intervention strategies early, such as educational and lifestyle modification programmes, including physical training regimes designed to address the high prevalence of CVD, musculoskeletal disorders, and complaints, and the low levels of physical fitness amongst the majority of firefighter and, thereby, attempt to reduce the elevated morbidity and mortalities rates in the fire services, globally.

## Figures and Tables

**Figure 1:** Bibliometric analysis of database search results.

**Figure 2:** Flowchart of the study selection.

**Figure 3:** Flow diagram illustrating the relationship between CVD risk factors, musculoskeletal health, physical fitness, and occupational performance in firefighters. (a) Indicates an unfit firefighter performing the stair climb test with much difficulty, and representing decreased occupational performance; (b) indicates a fit firefighter performing the stair climbtest with ease, representing optimal occupational performance. Black lines indicate cardiovascular disease risk factors; red lines indicates cardiovascular health and all related outcomes; blue lines indicate musculoskelatal health and all related outcomes; green lines indicate physical fitness and all related outcomes; purple lines indicate occupational performance and all related outcomes.

**Table 1:** Search strategy for PubMed.

Order	Search terms
#1	“firefighter” [MeSH] OR “fire and rescue personnel” [MeSH] OR “fire fighters” [MeSH] OR “fire fighter” [MeSH]
#2	“Cardiovascular system”[MeSH] OR (“cardiovascular”[All fields] AND “system”[All fields]) OR “cardiovascular system”[All fields] OR “cardiovascular”[All fields] OR “cardiovasculars”[All fields] OR “cardiovascular abnormalities”[MeSH] OR “cardiovascular health” OR “HRV”[All fields] OR “heart rate variability” [All fields] OR “Heart Rate
	“Interval” [All fields] OR “RR variability” [All fields] OR “cycle length variability” [All fields] OR “heart period variability” [All fields] OR “autonomic function” [All fields] OR “vagal control” [All fields] OR “lipid profile” [MeSH] OR “cholesterol” [MeSH] “diabetes” OR “blood glucose” OR “age” OR “obesity” OR “blood pressure” OR “blood glucose” OR “Diet” OR “eating habits” OR “eating culture”

#3	“muscular injury” (MeSH) OR (“musculoskeletal” [All fields] AND “system” [All fields]) OR “muscular pain” OR “chronic pain” OR “acute pain” “acute injury” OR “muscular health”

#4	“Physical fitness” [MeSH] OR “exercise” [All fields] OR “physical exertion” [All fields] OR “fitness” OR “body composition” [MeSH] OR “muscle” AND (“strength” OR “endurance” OR “flexibility” OR “power”) OR “cardiorespiratory”

#5	“work performance” [All fields] OR “endurance” [All fields] OR “fitness” [All fields] OR “performance” [MeSH] AND “work performance/classification” [MeSH] OR “occupational health” OR “employee health” [MeSH] OR “occupational performance” OR “work ability” OR “health, industrial” [MeSH] OR “industrial health” [MeSH] OR “occupational safety” [MeSH] OR “safety, occupational” [MeSH] “body composition” [MeSH] OR “muscle” AND (“strength” OR “endurance” OR “flexibility” OR “power”) OR “cardiorespiratory”

#6	#1 AND #2 OR #1 AND #3 OR #1 AND #4 OR #1 AND #2 AND #3 OR #1 AND #2 AND #4 OR #1 AND #3 AND #4 OR #1 AND #2 AND #3 AND #4 OR #1 AND #5 OR #2 AND #5

**Table 2:** Inclusion and exclusion criteria of the literature search.

Inclusion criteria	Exclusion criteria
(i) Studies involving firefighters, either career, part-time, or volunteer.	(i) Studies that did not include firefighters only (other emergency services and populations excluded).
(ii) Studies investigating the relationships between cardiovascular disease risk factors, musculoskeletal health/disorders/injuries, physical fitness metrics, and occupational performance.	(ii) Review studies.
(iii) Studies published after the year of 2000.	(iii) Intervention studies.
(iv) Quantitative or mixed methods studies.	(iv) Qualitative studies that do not include quantitative statistical analysis.
	(v) Languages other than English.
	(vi) Articles where full-text was not available.

**Table 3:** Search results from electronic databases.

Database	Search results
PubMed	807
Web of science	973
SCOPUS	823
Grey literature	4
Total	2607

**Table 4:** Relationship between CVD risk factors musculoskeletal health, physical fitness, and occupational performance (*n* = 46).

References	Year	Sample and setting	Study design (sampling)	Outcome
*Cardiovascular disease risk factors and musculoskeletal health (n* *=* *7)*				
Poston et al. [41]	2011	478 full-time male firefighters	Cross-sectional	(i) Age, BMI, smoking status, and general health were significant predictors of work injury (*p* < 0.001).
		USA		(ii) Firefighters categorised with class II and III obesity were significantly more likely to sustain injuries (OR: 4.89).
Jahnke et al. [22]	2013	347 full-time firefighters	Prospective cohort	(i) Obese firefighters were 5.2 times more likely to experience musculoskeletal injury.
		Kansas, Missouri, Iowa, Nebraska, North Dakota, South Dakota, Colorado, and Wyoming, US		(ii) Firefighters with central obesity were 2.8 times more likely to experience musculoskeletal injury.
Jahnke et al. [21]	2013	462 full-time firefighters	Cross-sectional	(i) Cigarette smokers were more likely to sustain injuries compared to nonsmokers.
		Kansas, Missouri, Iowa, Nebraska, North Dakota, South Dakota, Colorado, and Wyoming, US		
Gordon and Lariviere [42]	2014	252 full-time male and female firefighters	Cross-sectional	(i) Age (OR: 6.49) and years of experience (OR: 0.1) were significant predictors of injury.
		Ontario, Canada		
Jang et al. [43]	2016	392 full-time firefighters	Cross-sectional	(i) Age was a significant predictor of lumbar intervertebral disc degeneration (*p* < 0.05), regardless of core job description.
		Dongguk, Goyang, Korea		
Damrongsak et al. [44]	2017	298 male firefighters conveniently sampled	Cross-sectional	(i) Age (*p*=0.002), BMI (*χ*^2^ = 127.84, df = 4, *p* < 0.0001), current back pain, occupational stress, history of back pain were significant predictors of current back pain.
		Southeastern United States, USA		
Negm et al. [45]	2017	294 full-time firefighters	Cross-sectional	(i) Older (≥42 years) firefighters had significantly more severe lower-extremity disability and more severe back pain
		Hamilton, Trenholme, Canada		(ii) Older firefighters were significantly more likely to have multiple musculoskeletal disorders.
*Cardiovascular disease risk factors and physical fitness (n* *=* *17)*				
Donovan et al. [46]	2009	214 male firefighters	Cross-sectional	(i) Cardiorespiratory fitness was inversely related to metabolic abnormalities (*p* < 0.001).
		Colorado, USA		
Baur et al. [47]	2011	968 male firefighters,	Cross-sectional	(i) Metabolic equivalents (METs) were inversely related to diastolic blood pressure (DBP), body fat, triglycerides, low-density lipoprotein cholesterol (LDL-C) and total/high-density cholesterol (TC/HDL-C) ratio, and high-density lipoprotein cholesterol (HDL-C).
		USA		
Punakallio et al. [24]	2012	70 male firefighters aged 30 to 44 years	Longitudinal	(i) Increased weekly exercise reduced the decline in cardiorespiratory fitness.
		Finland		(ii) Regular smoking and more than 15 units of alcohol a week were significant predictors of a decline in cardiorespiratory fitness.
Baur et al. [48]	2012	1149 male firefighters, USA	Cross-sectional	(i) Cardiorespiratory fitness was inversely associated with ECG and autonomic exercise testing abnormalities before and after adjustment for age, BMI and metabolic syndrome.
Mayer et al. [49]	2012	83 full-time firefighters	Cross-sectional	(i) Back and core muscular endurance was 27% lower in obese firefighters. Back and core muscle endurance were related to obesity.
		Tampa, Florida, USA		(ii) Significant negative correlations were reported between back endurance and age (*p* < 0.05), BMI (*p* < 0.01), and BF% (*p* < 0.01), and between core endurance and BMI (*p* < 0.01), BF% (*p* < 0.01), and fat free mass (*p* < 0.05).
Poplin et al. [50]	2013	577–799 full-time firefighters	Longitudinal	(i) Age was a significant modifier of V̇O_2max_ (*p* < 0.001).
		Southwestern States, USA		
Kiss et al. [51]	2014	1225 firefighters	Cross-sectional	(i) Cardiorespiratory fitness was significantly related to age-group, body mass index (BMI) groups, and body fat percentage.
		East-Flanders Province, Belgium		
Walker et al. [52]	2014	73 full-time male firefighters, Australia	Cross-sectional	(i) Aging was significantly related to poor cardiorespiratory fitness (*p* < 0.05).
				(ii) Aging was related to a significant decrease in cardiorespiratory fitness between the 35–44 and 45–54-year age groups (*p* < 0.001).
Poplin et al. [53]	2015	799 full-time firefighters	Retrospective occupational cohort	(i) Age was negatively correlated with V̇O_2max_ (*r* = −0.368, *p* < 0.05), flexibility (*r* = −0.160, *p* < 0.05).
		Southwestern states, USA		(ii) BF% was negatively correlated with V̇O_2max_ (*r* = −0.448, *p* < 0.05), grip strength (*r* = −0.191, *p* < 0.05), and flexibility (*r* = −0.135, *p* < 0.05).
Seyedmehdi et al. [29]	2016	157 full-time male firefighters, Tehran	Cross-sectional	(i) Cardiorespiratory fitness (V̇O_2max_) was significantly correlated with age, BMI, cigarette smoking, physical activity, LDL-C, HDL-C, SBP, DBP, and heart rate (*p* ≤ 0.05).
Kirlin et al. [54]	2017	97 female firefighters, San Diego, USA	Cross-sectional	(i) Relative V̇O_2_, absolute V̇O_2_ and maximum METs were significantly associated with age.
Li et al. [55]	2018	294 full-time firefighters, Colorado, USA	Cross-sectional	(i) BF% (*p* < 0.01), estimated V̇O_2max_ (*p* < 0.05), metabolic syndrome (*p* < 0.05), and age group (*p* < 0.001) were significantly related to 10-year atherosclerotic cardiovascular disease risk.
Barry et al. [56]	2019	29 male full-time firefighters conveniently sampled, USA	Cross-sectional	(i) Waist circumference (WC) was a significant predictor of V̇O_2max_.
				(ii) More physically active firefighters had a higher V̇O_2max._
Espimoza et al. [57]	2019	76 volunteer male firefighters, Chile	Cross-sectional	(i) Age, BMI, WC, waist-to-hip ratio (WHR), BF% and fat mass was significantly correlated with V̇O_2max_.
				(ii) Resting heart rate (RHR), SBP, DBP, and blood glucose were significantly correlated with V̇O_2max_.
Porto et al. [58]	2019	64 full-time firefighters (38 on-duty and 26 off-duty), federal District (Brasilia), Brazil	Cross-sectional	(i) Cardiorespiratory fitness (V̇O_2max_) was positively correlated with overall cardiac autonomic function and higher parasympathetic activity (*p*=0.03).
Yang et al. [59]	2019	1562 full-time firefighters participated at baseline and 1104 of these firefighters participated at follow-up, Indiana, USA	Retrospective longitudinal cohort	(i) Age, BMI, SBP, DBP, total cholesterol (TC), LDL-C, triglycerides, glucose concentration, and smoking status were significantly different between push-up categories (upper body endurance).
Strauss et al. [8]	2021	97 full-time firefighters <60 years. Westphalia, Germany	Cross-sectional	(i) BMI, WC, BF%, and resting SBP, triglycerides, and total cholesterol values were significantly lower with increased cardiorespiratory fitness (V̇O_2max_) (*p* < 0.05, age-adjusted).
*Cardiovascular disease risk factors and occupational performance (n* *=* *6)*				
Airila et al. [60]	2012	403 male firefighters, Kuopio, Finland.	Longitudinal	(i) Age (*r* = −0.33, *p* < 0.01) and BMI (*r* = −0.15, *p* < 0.05) were negatively related to work ability, and cigarette smoking was negatively related to work demands (*r* = −0.10 *p* < 0.05), and physical exercise was positively related to work ability index (*r* = 0.015, *p* < 0.01) and work demands (*r* = 0.018, *p* < 0.01).
Walker et al. [52]	2014	73 full-time male firefighters, Australia	Cross-sectional	(i) Aging was significantly related to worse performance of simulated operational power testing tasks (*p* < 0.001).
				(ii) Hose-drag times significantly increased between 25–34 and 45–54 (*p* < 0.001) and 35–44 and 45–54 year age-groups (*p* < 0.001). Dummy-drag times significantly increased between 25–34 and 45–54 (*p* < 0.001), and 35–44 and 45–54-year age-groups (*p* < 0.001).
Firoozeh et al. [61]	2017	375 full time male firefighters, Tehran	Cross-sectional	(i) Age (*r* = -0.277, *p*=0.001), BMI (*r* = −0.187, *p*=0.001) and work experience (*r* = −0.281, *p*=0.001) were negatively correlated with work ability.
				(ii) Leisure time physical activity (*r* = 0.206, *p*=0.001) was related to work ability.
Phillips et al. [7]	2017	414 male firefighters, Alberta, Canada	Longitudinal	(i) The obese firefighting group had a significantly shorter treadmill time, lower relative V̇O_2max_ and absolute V̇O_2max_.
				(ii) The heaviest groups had significantly lower completion times for the hose drag, weighted sled pull, forcible entry, and victim rescue.
				(iii) The lightest firefighters had a significantly lower time for the ladder climb.
Nazari et al. [26]	2018	46 male and 3 female firefighters between the ages of 20–69 years, Canada	Secondary analysis	(i) Age and grip strength were significant predictors of hose drag and stair climb completion times (*p* < 0.05).
Saari et al. [62]	2020	74 full-time male firefighters were conveniently sampled, Kentucky, USA	Cross-sectional	(i) Older firefighters (≥37 years) had an 8.8% increase in completion time for the firefighting course.
				(ii) Age was positively correlated with course time (*r* = 0.297, *p*=0.017).
Xu et al. [63]	2020	20 full-time male firefighters, Southeast China	Cross-sectional	(i) High BF% was associated with poor performance in ability tests.
Norris et al. [64]	2021	19 full-time male firefighters, Texas, USA	Cross-sectional	(i) Age and fat mass were significant predictors of work efficiency.
*Musculoskeletal health and physical fitness (n = 5)*				
Wynn and Hawdon [65]	2012	Firefighter recruits with minimum cardiorespiratory fitness standard (398 full-time and 48 part-time recruits) and without fitness standard (198 full-time and 206 part-time subjects). Northern England	Cohort	(i) Injury-related restrictions were more likely where no cardiorespiratory fitness standard was applied.
				(ii) Firefighters with a higher V̇O_2max_ correlated with a lower incidence of injuries (*p* < 0.01)
Butler et al. [66]	2013	108 trainee firefighters, Orange County, USA	Cohort	(i) Three functional movement screening (FMS) movements were significant predictors of injury i.e., the sit-and-reach (OR: 1.24), the deep-squat (OR: 1.21), and the push-up (OR: 1.30).
Jahnke et al. [21]	2013	462 full-time firefighters, Kansas, Missouri, Iowa, Nebraska, North Dakota, South Dakota, Colorado, and Wyoming, USA	Cross-sectional	(i) Injuries were 4.6 times more likely to be sustained when firefighters regularly exercised, while on duty. Increased V̇O_2max_ (OR: 1.06) and strength (OR: 4.03) were significantly associated with injury while exercising or training.
Poplin et al. [50]	2013	577–799 full-time firefighters, Southwestern States, USA	Longitudinal	(i) Firefighters in the lowest fitness category (V̇O_2max_ < 43 mL·kg^−1^·min^−1^) were 2.2 times more likely to sustain injury than firefighters in the highest fitness level category (V̇O_2max_ > 48 mL·kg^−1^·min^−1^).
				(ii) A V̇O_2max_ between 43 and 48 mL·kg^−1^·min^−1^ were 1.38 times more likely to incur injury.
				(iii) Improving relative aerobic capacity by one metabolic equivalent reduced the risk of injury by 14%.
Poplin et al. [53]	2015	799 full-time firefighters, Southwestern States, USA	Retrospective occupational cohort	(i) Firefighters with lower cardiorespiratory fitness were at increased risk of injury.
				(ii) The risk of injury was 1.82 times more likely for the least fit firefighters.
				(iii) When restricted to sprains and strains, the risk of injury increased to 2.90.
*Musculoskeletal health and occupational performance (n* *=* *5)*				
Punakallio et al. [67]	2014	411 full-time male firefighters, Helsinki, Finland	Longitudinal	(i) Musculoskeletal pain (MSP) in more than one site diminished work ability.
				(ii) Low back pain (OR = 1.9) forearm and hands pain (OR = 1.9) predicted diminished work ability
				(iii) Participants who were on disability pension were older, more often had poor work ability, and had slightly more MSP at baseline.
				(iv) Average-(OR: 3.1)-to-high (5.3) physical workload was a significant risk factor for retiring on disability pension.
Kodom-Weredu [68]	2018	320 full-time firefighters	Cross-sectional	(i) Work-related musculoskeletal disorders (WMSD) were significantly related to work demands (*r* = 0.023) and task characteristics (*r* = 0.026). Work demands (*β* = 0.226, *p* < 0.01) and task characteristics (*β* = 0.214, *p* < 0.01) were significant predictors of WRMSDs.
		The greater Accra region of Ghana		
MacDermid et al. [40]	2019	293 full-time male and female firefighters	Cross-sectional	(i) Firefighters who reported moderate-severe muscle and joint problems took 10 seconds longer to perform the stair climb, but were not statistically significant.
		Hamilton, Ontario, Canada		
Saremi et al. [69]	2019	250 full-time firefighters	Cross-sectional	(i) Work ability index had negative correlation with discomfort in the wrists (*r* = –0.170, *p*=0.007), legs (*r* = –0.129, *p*=0.042), and ankles (*r* = –0.176, *p*=0.005.
		Tehran (North, South, East, and West)		
Nazari et al. [39]	2020	325 full-time firefighters	Cross-sectional survey	(i) Firefighters with spinal pain experienced significantly more output limitation. Firefighters above 45 years experienced more physical work limitations. The number of musculoskeletal pain sites, age, and years of service predicted occupational output and work limitations.
		Hamilton, Ontario, Canada		
*Physical fitness and occupational performance (n* *=* *11)*				
von Heimburg et al. [70]	2006	13 full-time male firefighters aged between 24 and 56 years.	Cross-sectional	(i) V̇O_2max_ was a significant predictor of simulation performance time. Better work performance was related to firefighters who were stronger, heavier, and taller.
		Nord-Trøndelag County, Norway		
Elsner and Kolkhorst [84]	2008	20 full-time male firefighters	Cross-sectional	(i) There was a moderately strong inverse relationship between the average V̇O_2max_ during the firefighting simulation protocol and performance time.
		San Diego, USA		
Sheaff et al. [72]	2010	33 full time firefighters, male (26) and female (7) aged between 18 and 45 years	Cross-sectional	(i) V̇O_2max_, upper body strength, grip strength, and the HR response to stair climbing were significantly related to better performance on the candidate physical ability test (*p* < 0.01). Absolute V̇O_2max_ predicted candidate physical ability test performance (*p*=0.001).
		Baltimore, Washington, USA		
Michaelides et al. [73]	2011	90 full-time firefighters	Cross-sectional	(i) Ability test (AT) completion time was associated with abdominal strength (*p* < 0.01), relative power (*p* < 0.01), upper-body muscular endurance and upper-body strength (*p* < 0.01). Poor performance on the AT was associated with high resting heart rate (*p* < 0.01), high BMI (*p* < 0.01), high BF% (*p* < 0.01), aging (*p* < 0.01), and high WC (*p* < 0.01).
		Arkansas, USA		
Heimburg et al. [74]	2013	63 full-time firefighters.	Cross-sectional	(i) Firefighters with higher a V̇O_2max_ who were stronger completed the simulation protocol faster (*p* < 0.05). Some firefighters with below average strength were among the quickest, indicating that a minimal strength was needed to perform well, and strength beyond that point did not improve performance times.
		Trondheim, Norway.		
Kleinberg et al. [75]	2016	46 full-time male firefighters aged 24 to 50 years	Cross-sectional	(i) Quadriceps muscle strength was significantly associated with stair climb time (*r* = 20.492, *p*=0.001), and remained significant after adjustment for age and BMI.
		North Carolina, USA		
Siddal et al. [76]	2018	68 (63 male; 5 female) full-time firefighters	Cross-sectional	(i) Age, sex, height and/or lean mass were not significant predictors of the firefighter simulation test (FFST) performance time. The strongest predictor of FFST time was absolute V̇O_2_ and fat mass.
		Bath, England, United Kingdom		
Nazari et al. [26]	2018	46 male and 3 female firefighters between the ages of 20–69 years.	Secondary analysis	(i) Grip strength and lower body strength were significant predictors of hose drag and stair climb completion times (*p* < 0.05), respectively.
		Canada		
Skinner et al. [77]	2020	42 male aviation rescue firefighters (ARFF)	Cross-sectional	(i) V̇O_2max_ (*p* < 0.001), anaerobic step test (*p* < 0.001), height (*p*=0.038) and lean mass (*p*=0.005) were inversely correlated with ARFF emergency protocol simulation performance time. Slower performance time was associated with higher fat mass (*p*=0.043) and BF% (*p*=0.001). Muscular strength, muscular endurance and flexibility were not related to performance on the simulated ARFF emergency protocol.
		Queensland, Australia		
Xu et al. [63]	2020	20 full-time male firefighters	Cross-sectional	(i) High BF% was associated with poor performance in ability tests, V̇O_2max_ was associated with increased performance, and upper and lower body muscular power were both inversely related to firefighter ability test completion time.
		Southeast China		
Norris et al. [64]	2021	19 full-time male firefighters	Cross-sectional	(i) Experience, jump height, inverted row endurance, relative bench and squat strength, and relative V̇O_2_ were significant predictors of work efficiency (*p* < 0.05).
		Texas, USA		

*Note*. Studies that were included were categorised chronologically. Few studies compared variables in more than one relationship and, therefore, few studies are repeated in the table.

## Data Availability

This is a review article and, therefore, no direct data will be available.
